# *KRAS* mutational status analysis of peripheral blood isolated circulating tumor cells in metastatic colorectal patients

**DOI:** 10.3892/ol.2013.1544

**Published:** 2013-08-23

**Authors:** CRISTINA GUTIÉRREZ, JAVIER RODRIGUEZ, ANA PATIÑO-GARCÍA, JESÚS GARCÍA-FONCILLAS, JOSEFA SALGADO

**Affiliations:** 1 Clinical Genetics Unit, University Clinic of Navarra, Pamplona, Navarra 31008, Spain; 2 Department of Oncology, University Clinic of Navarra, Pamplona, Navarra 31008, Spain; 3 Jiménez Díaz Foundation, Madrid 28040, Spain

**Keywords:** circulating tumor cells, metastatic colorectal cancer, *KRAS* gene, peripheral blood, inmunomagnetic labeling

## Abstract

The present study describes an optimized method for isolating peripheral blood circulating tumor cells (CTCs) and performing *KRAS* mutation analysis. The approach combines isolation of peripheral blood mononuclear cells and immunomagnetic labeling with CD45 and CD326 human microbeads with KRAS analysis performed with a Therascreen KRAS kit by quantitative PCR. *KRAS* mutations were detected in the CTCs of patients with metastatic colorectal cancer (mCRC). CTCs may represent an alternative to invasive procedures and their analysis may be representative of the current disease status of the patient. This proposed analysis may be performed in a daily clinical practice.

## Introduction

Colorectal cancer (CRC) is one of the most significant worldwide public health problems (1). During the natural course of the disease, ~50% of patients may develop metastasis and up to 25% of these present with metastatic disease at the moment of diagnosis. Advances in the treatment of metastatic colorectal cancer (mCRC) include the development of new antitumoral agents, including epidermal growth factor receptor-targeted monoclonal antibodies (EGFR-mAbs) and tyrosine kinase inhibitors, and the use of biomarkers. The *KRAS* mutational status is currently the only biomarker that is predictive of the response to therapy using EGFR-mAbs that have been validated for clinical practice in mCRC and recommended by the National Comprehensive Cancer Network (NCCN) 2012 Guidelines (version 1, 2012) (2,3). However, not all mCRC patients with wild-type *KRAS* respond to EGFR-mAb treatment, which may be due to alterations in other genes, including *BRAF*, *PIK3CA* and *PTEN*(4,5). Furthermore, numerous studies have shown discordance in the *KRAS* mutational status between the primary tumor and the metastatic lesions (6–8). Thus, the study of *KRAS* in metastases may have clinical relevance and may, at least partly, explain the resistance to EGFR-mAbs in patients with *KRAS* wild-type primary tumors. Metastasis involves the concept of circulating tumor cells (CTCs) that are associated with the colonization of distant organs. Since the study by Ashworth in 1869, in which malignant cells that were similar to the primary tumor were identified to circulate in the peripheral blood (9), increased efforts, particularly in recent years, have focused on the development of reliable methods for the enrichment and identification of CTCs (10–12). The present study describes an easy, affordable procedure using magnetic labeling that allows the isolation of an enriched CTC fraction from peripheral blood and, furthermore, the analysis of the *KRAS* mutational status of the CTCs. A comparison between the *KRAS* mutational status in CTCs and the corresponding tumor tissue was performed.

## Materials and methods

### Patients

A total of 23 mCRC patients who were in remission or whose primary tumor *KRAS* mutational status was available in the patient clinical records were selected for this study. Ethylenediaminetetraacetic acid (EDTA)-anticoagulated peripheral blood (10 ml) was obtained from each patient, all of who exhibited disease progression. This study was approved by the ethics committee of the University Clinic of Navarra. All the participants provided their informed consent prior to blood sample extraction.

### Isolation of peripheral blood mononuclear cells (PBMCs; time, 1.5 h)

When working with anticoagulated peripheral blood, PBMCs should be isolated using density gradient centrifugation. Ficoll-Paque™ Plus was used for this purpose (17-1440-03; GE Healthcare, Buckinghamshire, UK). The blood samples were diluted with saline serum (ratio, 1:1) and gently added on the top of the Ficoll-Paque Plus medium (ratio, 2/3 blood:1/3 Ficoll) taking care not to mix the two layers. Following centrifugation for 20 min at 400 × g, the PBMCs that were located at the interface layer were collected by inserting the pipette directly through the plasma (alternatively, the upper plasma layer may be removed and the PBMCs may be collected). The PBMCs were washed twice with saline serum and centrifuged for 8 min at 300 × g. Buffer A was added to the PBMCs, which were then centrifuged at 200 × g for 10–15 min. Buffer A consisted of phosphate-buffered saline (PBS; pH 7.2), 0.5% bovine serum albumin (BSA) and 2 mM EDTA). This step was repeated twice.

### Enrichment of circulating tumor cells (time, 2 h)

CD45 Human MicroBeads (130-045-801; Miltenyi Biotec GmbH, Bergisch Gladbach, Germany) were used for the enrichment of the epithelial tumor cells from the peripheral blood by the depletion of the CD45^+^ cells. The cell number from the previous step was measured and following centrifugation at 300 × g for 10 min and complete aspiration of the supernatant, 80 μl buffer A and 20 μl CD45 MicroBeads per 10^7^ total cells were added, mixed and refrigerated (4–8°C) for 15 min. Following a wash step with 2 ml buffer A per 10^7^ cells (300 × g for 10 min), 500 μl buffer A was added (up to 10^8^ cells). The cell suspension was loaded onto a separator column that was placed in a magnet (MiniMACS Starting kit; Miltenyi Biotec). The magnetically-labeled CD45^+^ cells were retained within the column. The unlabeled cell fraction (CD45^−^ fraction) that was enriched in the epithelial tumor cells ran through.

### CD326 epithelial cell adhesion molecule (EpCAM) Human MicroBeads are used for the enrichment of epithelial tumor cells

The cell number from the CD45^−^ fraction that was obtained in the previous step was measured and following centrifugation at 300 × g for 10 min and complete aspiration of the supernatant, 300 μl buffer A and 100 μl FcR reagent (120-000-442; Miltenyi Biotec) per 5×10^7^ total cells were added and mixed. A total of 100 μl CD326 Microbeads were added per 5×10^7^ total cells, mixed well and refrigerated at 4–8°C for 30 min. Following a wash step with 5–10 ml buffer A per 5×10^7^ cells (300 × g for 10 min), 500 μl buffer A was added up to 10^8^ cells). The cell suspension was loaded onto a separator column placed in a magnet (MiniMACS Starting kit; Miltenyi Biotec). Subsequent to the labeling and separating procedures, three cell fractions were obtained, CD45^+^, CD45^−^/CD326^−^ and CD45^−^/CD326^+^. A schematic of the procedure is shown in Fig. 1.

### DNA purification and quantification (time, 1 h)

The QIAamp^®^ Mini kit (51101; Qiagen GmbH, Hilden, Germany) was used for DNA purification from the cell fractions that were obtained previously. The procedure was performed as described in the QIAamp Mini kit instructions. DNA quantification was performed using the NaNoDrop-2000/2000c Spectrophotometer (Thermo Fisher Scientific Inc., Waltham, MA, USA), following the manufacturer’s instructions.

### KRAS mutational status analysis (time, 2.5 h)

All DNA was analyzed for a set of seven *KRAS* point mutations, 12-Ala, Asp, Arg, Cys, Ser, Val and 13-Asp, using the Therascreen KRAS kit (870011; Qiagen GmbH). The analysis was performed on a quantitative PCR instrument (Rotor-Gen Q; Qiagen GmbH).

## Results and discussion

Blood samples were studied from 23 mCRC patients whose primary tumor *KRAS* mutational status was available. Following the enrichment of the CTCs, three fractions were obtained, CD45^+^, CD45^−^/CD326^−^ and CD45^−^/CD326^+^. The *KRAS* Mutation kit detected seven specific *KRAS* mutations using a region of the *KRAS* exon-4 as a control. The CD45^+^ cell fraction contained mainly leukocytes, thus, a signal appeared in the control assay that corresponds to the *KRAS* exon-4, but no *KRAS* mutation was detectable, since somatic mutations were only present in the fraction that contains the CTCs, if detectable. The CD45^−^/CD326^−^ and CD45^−^/CD326^+^ cell fractions exhibited a signal of the *KRAS* exon-4 control due possibly to the residual mononuclear cells; however, the amplification signal appeared at a higher cycle compared with the corresponding CD45^+^ since the expected mononuclear cells amount was low. The CTCs were identified in the CD45^−^/CD326^+^ cell fraction and, therefore, the *KRAS* mutations, if detectable by the kit, appear in this fraction. The present study identified a correspondence between the primary tumor-*KRAS* status and the CTC-*KRAS* status in 17 patients (15 wild-type and two mutated). In five cases, the tumor-*KRAS* mutation was not detected in the CTCs. In those patients, a low concentration of CTCs explained the results as their DNA concentration was below the kit detection limits. Notably, another discrepancy was identified in one patient (case CR6), who demonstrated a *KRAS* wild-type in the primary tumor and a *KRAS*-12Ala mutation in the CTC enriched cell fraction (Fig. 2). In this case, another scenario should be proposed. It is known that in a minority of cases (5–10%) the *KRAS* mutational status is heterogeneous and may vary between the primary tumor and the metastasis (13). In a recent study, Bossard *et al* defined a KRAS mutational mosaicism, with 4 out of 18 patients showing *KRAS* status discordances between the primary colorectal cancer and the metastasis (14). The biological significance of this mosaicism is unclear, but indicates diverse metastatic potentials in various populations of tumor cells and/or the acquirement of mutations during or following metastasis. Bouchahda *et al* proposed that *KRAS* mutations may be acquired late during the metastatic phase of colorectal cancer more frequently than currently recognized (15). Furthermore, since CTCs may be considered as an intermediate step in colonization, their metastatic potential depends on a number of genetic abnormalities that may include the acquisition of a *KRAS* mutation. Therefore, the CTC-*KRAS*-Ala mutation that was identified in a patient from the present study may lead to an improved adaptation to adverse conditions, migration and colonization of distant tissues. By the end of the present study, the CR6 patient developed hepatic metastasis (tissue from metastases not available) and a change from anti-EGFR to Irinotecan-based treatment was considered. Future studies examining large series and examining *KRAS*, *BRAF*, *PTEN* and *PI3K* may provide valuable insight into the carcinogenesis and metastasizing patterns of mCRC, thus guiding treatment options for patients.

In summary, the present study indicated that the isolation and analysis of CTCs from the peripheral blood of mCRC patients, using a minimally invasive, relatively economical and optimized method, may have high clinical relevance. There are limitations to the procedure, since during epithelial to mesenchymal transition, the expression of epithelial markers on CTCs, such as EpCAM may be downregulated and become undetectable (16). CTC studies represent an alternative to invasive procedures and their analysis may become a prognostic factor, acting as a ‘liquid biopsy’. CTCs are able to survive chemotherapy and may indicate a lack of therapeutic efficacy, allowing the early end of ineffective treatments and providing a representation of the current disease status of the patient.

## Figures and Tables

**Figure 1:** Schematic procedure of the *KRAS* mutational status analysis of peripheral blood isolated CTCs in mCRC patients. PCR, polymerase chain reaction; CTCs, circulating tumour cells; mCRC, metastatic colorectal cancer.

**Figure 2:** Image of the CTC-*KRAS* mutational status for patient CR6. The CD45^+^ cell fraction (mainly leukocytes) provides a positive signal for the control assay corresponding to *KRAS* exon-4. The CD45^−^/CD326^−^ cell fraction exhibits a positive signal of the control assay corresponding to *KRAS* exon-4. The CD45^−^/CD326^+^ cell fraction exhibits a positive signal of the control assay corresponding to *KRAS* exon-4 and a signal for the *KRAS*-12Ala mutation. CTC, circulating tumour cell.
